# A Multiscale Clustering Approach for Non-IID Nominal Data

**DOI:** 10.1155/2021/8993543

**Published:** 2021-10-11

**Authors:** Runzi Chen, Shuliang Zhao, Zhenzhen Tian

**Affiliations:** ^1^School of Mathematical Sciences, Hebei Normal University, Shijiazhuang 050024, China; ^2^College of Computer and Cyber Security, Hebei Normal University, Shijiazhuang 050024, China; ^3^Hebei Provincial Key Laboratory of Network and Information Security, Shijiazhuang 050024, China; ^4^Hebei Provincial Engineering Research Center for Supply Chain Big Data Analytics & Data Security, Shijiazhuang 050024, China; ^5^State Grid Xingtai Electric Power Supply Company, Xingtai 054000, China

## Abstract

Multiscale brings great benefits for people to observe objects or problems from different perspectives. Multiscale clustering has been widely studied in various disciplines. However, most of the research studies are only for the numerical dataset, which is a lack of research on the clustering of nominal dataset, especially the data are nonindependent and identically distributed (Non-IID). Aiming at the current research situation, this paper proposes a multiscale clustering framework based on Non-IID nominal data. Firstly, the benchmark-scale dataset is clustered based on coupled metric similarity measure. Secondly, it is proposed to transform the clustering results from benchmark scale to target scale that the two algorithms are named upscaling based on single chain and downscaling based on Lanczos kernel, respectively. Finally, experiments are performed using five public datasets and one real dataset of the Hebei province of China. The results showed that the method can provide us not only competitive performance but also reduce computational cost.

## 1. Introduction

Clustering is one of the vital data mining and machine learning techniques, which aims to group similar objects into the same cluster and separate dissimilar objects into different clusters [1]. It is so prominent and recently attracted significant attention of researchers and practitioners from different domains of science and engineering [2]. Thousands of papers had been published [3–6]. However, these investigations only concentrated on clustering at a single perspective.

The scale can be equivalent to the following concept: generic concept, level of abstraction, or perspective of observation; the same problem or system can be perceived at different scales based on particular needs [2]. That is called multiscale phenomena and has been widely applied to the academic fields, such as geoscience [3, 4] and mathematics [5]. Based on the clustering for distribution of scapularis nymphs at different spatial scales of lyme disease occurrence areas in southern Quebec, Canada, reference [6] helps people understand the change of risk and take corresponding measures. In [7], an average linkage hierarchical clustering algorithm was proposed through the regionalization algorithm to identify uniform rainfall areas in nonstationary precipitation time series based on multiscale self-lifting sampling. The authors in [8] proposed a multiscale Gaussian kernel-induced fuzzy C-means algorithm to segment lesions and determine the edges of lesions.

From the current research situation, multiscale clustering has been widely studied in various disciplines. However, from the analysis of the attribute type of data, most of the research studies are only for the numerical dataset, the quantitative analysis, and prediction of the data, but there is very little qualitative analysis about nominal dataset. Most of the datasets use characters to represent attribute values and do not have the properties of numbers. Even if they are represented by numbers (integers), they should be symbols and cannot be analyzed quantitatively. To study the nominal dataset, not only the complex data characteristics need to be obtained but also the proposed method needs to have some flexibility.

The main contributions of this paper are as follows: (1) a multiscale clustering approach for Non-IID nominal data is proposed by introducing unsupervised coupling metric similarity; (2) combined with the scale-transformation theory and the idea of condensed hierarchical clustering, a scale calculation method based on a single chain is proposed to transform the clustering results from benchmark scale to target scale; and (3) combining the scale-transformation theory with Lanczos interpolation idea and based on the split hierarchical clustering idea, the Lanczos kernel-based downscaling algorithm was proposed to carry out multiscale clustering for the Non-IDD nominal datasets.

The rest of this paper is organized as follows.  Section 2 discusses the related work. Some definitions are reviewed briefly in Section 3. The framework of multiscale clustering is designed in Section 4.  Section 5 details the comparison experiments. The conclusion and some future research directions are given in Section 6.

## 2. Related Work

Clustering has attracted more and more attention from researchers and can be applied to many fields, such as time series analysis [9, 10], brain-computer interface [11–15], epilepsy [16, 17], and sleep staging [18, 19]. Clustering usually requires that the number of “classes” to be set in advance, and then the dataset is divided into each “class” according to the specific partitioning algorithm. The partitioning method assigns a dataset into *k* clusters such that each cluster must contain at least one element. The k-means algorithm proposed by MacQueen in 1967 is the most classical representation of the partitioning method [20], and that is one of the best-known and simplest clustering algorithms [21]. Frey and Dueck in 2007 proposed the “affinity propagation (AP)” algorithm [22]. Different from previous clustering algorithms, this algorithm does not need to determine the clustering center in advance but uses a N-order square matrix to store the relationship between data and performs iterative clustering on this square matrix with obvious results. In 2013, Kawano et al. proposed a greedy clustering algorithm based on *k* members and applied it to collaborative filtering tasks [23]. In 2015, Agarwal et al. proposed the improved k-means algorithm k-means ++, which is as decentralized as possible in the selection of centroid, and the clustering effect is significantly improved [24]. Spectral clustering [25] originates from graph theory. Data are regarded as vertices in the graph, and the relationship between data is regarded as edges in the graph. The graph is divided into several subgraphs by “graph cutting” technology, and the subgraphs correspond to clusters in the clustering. The common feature of these algorithms is that they can only handle numerical data. For the clustering problem of nominal data, Huang was inspired by the k-means algorithm and proposed the k-modes algorithm [26] for the first time in 1998. This algorithm adopted a new way of measuring object similarity to partition data objects. In 2018, Nguyen et al. improved the k-modes algorithm [27] and used the privacy protection mechanism to solve the problem of transparent data input.

In 2014, Saffarzadeh et al. used the multiscale linear algorithm to analyze retinal images to determine whether eye lesions occurred [28]. In 2015, Lim et al. applied the multiscale spectrum clustering algorithm in the field of geosciences to improve the reliability of earthquake prediction [29]. In 2016, Parisot et al. applied multispectral clustering to the medical field to improve the efficiency and accuracy of magnetic resonance imaging [30]. In 2018, Ripoche et al. investigated the distribution of lyme disease at three different spatial scales in southern Quebec, Canada, and the density of pupae in different woodlands and in different plots and sections of the same woodlands, to provide guidance on the understanding and prevention of lyme disease [6]. Vu et al. developed a new multithreaded tool, fMLC, and addressed the problem of clustering large-scale DNA sequences [31]. A multilevel clustering for star/galaxy separation was designed in 2016, consisting of three phases: coarsening clustering, representative data clustering, and merging [32]. In 2019, Zunic et al. proposed a multilevel clustering algorithm that is used on the Internal Banking Payment System in a bank of Bosnia and Herzegovina and explained how the parameters affect the results and execution time in the algorithm [33]. These all algorithms aim to a specific application and solve the corresponding problems. On the premise that the clustering results of small-scale data sets have been obtained, Chen et al. [34] proposed a method named SUCC to solve the clustering for large-scale data. We will propose a multiscale clustering approach for Non-IID nominal data.

In clustering, we need to evaluate the dissimilarity among objects by using distance measure [35]. Minkowski distance is the most commonly used measure for numerical data. The most popular distance measure is Euclidean distance, another well-known measure is the Manhattan distance, and they are all special cases of Minkowski distance. The dissimilarity between two binary attributes is computing a dissimilarity matrix from the given binary data. The above measurement methods are mainly for numerical data, and quantitative processing and analysis are carried out. However, there are also nonnumerical attribute values of data, also known as nominal data. At present, there are few studies on qualitative analysis of nominal data, especially the data are Non-IID. Couple metric similarity (CMS) [36] is good for measuring the distance of Non-IID nominal data.

## 3. Preliminaries

To facilitate the discussion in the remainder of this paper, CMS is reviewed briefly in this section. CMS measures the similarity of two objects by capturing both the intra- and inter-attribute coupling relations of objects, where the former characterizes the coupling similarity between the frequency distribution and the value of attribute and the latter aggregates attribute dependencies between different attribute values relationship by considering the intersection of the condition attribute values co-occurrence probability of the different characteristics [36].

**Definition 1 .**

(intra-attribute similarity). The intra-attribute similarity between two objects *A* and *B* on attribute *j* is *S*_Ia_ (*A*_j_, *B*_j_) and is defined as follows:

(1) $$\begin{array}{c} S_{Ia}\left(A_{j},B_{j}\right)=\left\{\begin{array}{cc} 1, & A_{j}=B_{j},\\ \frac{\log\;p\cdot \;\log\;q}{\log\left(p\cdot \;q\right)+\log\;p\;\cdot \;\log\;q}, & \text{others,} \end{array}\right. \end{array}$$

where *p*=|*N*(*A*_*j*_)|+1, *q*=|*N*(*B*_*j*_)|+1, *A*_*j*_ represents the value of object *A* on attribute *j*, *B*_*j*_ represents the value of object *B* on attribute *j*, *N*(*A*_*j*_) represents is the set of objects whose values of attribute are *A*_*j*_, and |•| represents the number of the set.

**Definition 2 .**

(inter-attribute similarity). The inter-attribute similarity between two values of attribute *A*_*j*_ and *B*_*j*_ on attribute *j* with other attributes is *S*_Ie_ (*A*_j_, *B*_j_) and is defined as follows:

(2) $$\begin{array}{c} S_{Ie}\left(A_{j},B_{j}\right)=\overset{d}{\underset{k=1,k\neq j}{\sum }}r_{k|j}S_{k|j}\left(A_{j},B_{j}\right), \end{array}$$

where *d* represents the number of attributes in dataset, *r*_*k|j*_ is the weight of each attribute *k* to attribute *j*, and *S*_*k|j*_(*A*_*j*_, *B*_*j*_) represents the inter-attribute similarity candidates with attribute *k* and is defined as follows:

(3) $$\begin{array}{c} S_{k|j}\left(A_{j},B_{j}\right)=\left\{\begin{array}{cc} 1, & A_{j}=B_{j},\\ \frac{M}{2M-Q}, & \text{others,} \end{array}\right. \end{array}$$

where

(4) $$\begin{array}{c} M=\overset{\left|W_{k}\right|}{\underset{i=1}{\sum }}\max\left(\frac{\left|N\left(W_{k}^{i},A_{j}\right)\right|}{\left|N\left(A_{j}\right)\right|},\frac{\left|N\left(W_{k}^{i},B_{j}\right)\right|}{\left|N\left(B_{j}\right)\right|}\right),\\ Q=\overset{\left|W_{k}\right|}{\underset{i=1}{\sum }}\min\left(\frac{\left|N\left(W_{k}^{i},A_{j}\right)\right|}{\left|N\left(A_{j}\right)\right|},\frac{\left|N\left(W_{k}^{i},B_{j}\right)\right|}{\left|N\left(B_{j}\right)\right|}\right), \end{array}$$

*W*_*k*_=*V*_*k*_^*N*(*A*_*j*_)^∩ *V*_*k*_^*N*(*B*_*j*_)^, where *V*_*k*_^*N*(*A*_*j*_)^ is the set of values of attribute *k* for all objects in *N*(*A*_*j*_) and *W*_*k*_ consists of those attribute values of attribute *k* which co-occur with both *A*_*j*_ and *B*_*j*_, *W*_*k*_^*i*^ is the ith element of *W*_*k*_.

**Definition 3 .**

(coupled metric similarity). The coupled metric similarity (CMS) between two objects *A* and *B* is *S*(*A*, *B*) and is defined as follows:

(5) $$\begin{array}{c} S\left(A,B\right)=\overset{d}{\underset{j=1}{\sum }}\beta_{j}S_{j}\left(A_{j},B_{j}\right), \end{array}$$

where *β*_*j*_ represents the weight of the coupled metric attribute value similarity of the an attribute *j* and *S*_*j*_(*A*_*j*_, *B*_*j*_) is defined as follows:

(6) $$\begin{array}{c} S_{j}\left(A_{j},B_{j}\right)=\frac{1}{\alpha \left(1/S_{Ie}\left(A_{j},B_{j}\right)\right)+\left(1-\alpha \right)\left(1/S_{Ia}\left(A_{j},B_{j}\right)\right)}, \end{array}$$

where *α* is the weighted harmonic mean of inter-attribute similarity and intra-attribute similarity. Different *α* reflects the different proportions of the intra-attribute similarity and inter-attribute similarity in forming the overall object similarity.

Throughout in this paper, we use CMS to measure the similarity of two objects.

## 4. Proposed Framework

The multiscale clustering framework proposed in this paper is shown in Figure 1. Instead of directly clustering on all scale datasets, this method first selects the best scale dataset that is named benchmark-scale dataset, then calls the classical mining algorithm on the benchmark-scale dataset to get the clustering results, and finally decides to push the clustering results up or down according to the relationship between the target scale and the benchmark scale. From this framework, it can be seen that the core of multiscale clustering is the benchmark-scale dataset clustering and the push up and push down of the clustering results of the benchmark-scale dataset. We design three algorithms to implement the framework.

Firstly, according to the probability density discretization method [37], the properties of the representational scale are divided into multiple scales by the probability density. Secondly, the optimal scale is determined according to the attenuation of the information entropy of each scale [38] and clustering on benchmark-scale dataset by using the spectral method. Details of Algorithm 1 are as follows. We calculate the distance between every pair sample in the benchmark-scale dataset by using CMS and construct the similarity matrix, where 1 ≤ *α*, *β* ≤ *ij*. (line 5). The Laplacian matrix be calculated in line 5–10. The value and vector are computed in line 11, where *N* is the number of cluster and set in advance. The core and label of cluster are spliced to form Rcenter (line 14).

After the clustering benchmark-scale dataset is completed, the cluster center of big-scale dataset can be deduced from the cluster center of the benchmark-scale dataset. In this paper, inspired by the idea of condensed hierarchical clustering, an upscaling algorithm based on CMS (UACMS) is proposed (line 2–4). Its basic ideas are as follows: each cluster center of the benchmark scale was taken as a cluster, and the CMS was distance measured, and the two nearest clusters were merged into one until the termination condition was reached (line 5–9). The specific process is as Algorithm 2.

The downscaling algorithm based on Lanczos (DSAL) obtains the cluster center of the small-scale dataset from the cluster center of the benchmark-scale dataset, and the process is exactly opposite to UACMS in Algorithm 3. That is, its principle is to adopt top-down thinking. Firstly, all the benchmark-scale cluster centers are regarded as a cluster, and Lanczos kernel function is used to calculate the weight of each cluster to generate new cluster centers (line 1). Then, more and smaller clusters are obtained according to the coupling similarity between them until the termination condition is met (line 2–5).

## 5. Performance Evaluations

In this section, we compare our method with classical methods: k-modes and the spectral clustering that are based on 5 measures (CMS, HM [39], OF, IOF, and Eskin [40]) on 6 datasets. The clustering evaluation index includes Normalized Mutual Information (NMI) [41], F-score [42], which belongs to external index score, and Mean Squared Error (MSE) [43, 44], which belongs to internal indicators, this section will use these three indicators to evaluate the accuracy of the proposed algorithm, and it also demonstrates the runtime advantage of the proposed algorithm.

### 5.1. Data and Experimental Settings

In order to verify the validity and feasibility of the framework and algorithm proposed in this paper, Kaggle and UCI public datasets (Zoo, Soybeanlarge, Dermatology, BreastCancer, and Titanic) and real datasets (renkou for short) were used for experimental verification, as shown in Table 1. To facilitate description, the datasets Soybeanlarge, Dermatology, and BreastCancer are represented by Sol, Der, and BrC, respectively, in this section. Our program has been implemented with Python and performed on a computer with a Inter(R) Core (TM) i7-3770 4-Core 3.4 GHz CPU, 8 GB RAM, and the windows 10 × 64 Home operating system.

### 5.2. Upscaling

The NMI values of the algorithm UACMS in this paper and the six comparison algorithms on each dataset are shown in Figure 2. It can be seen from the figure that the OF's NMI value is basically the smallest in each dataset, and the NMI value of the algorithm UACMS is the highest, except for BrC and Titanic. The main reason is that the relationship between the element attributes of the two datasets is complex. It is not easy to reflect this complex relationship by adjusting the parameters that restrict the weight of the relationship intra-attributes and the relationship inter-attributes of objects, which is also a challenge faced with the algorithm. Of course, UACMS performs well on Der, renkou, and other datasets. In general, the NMI value of the algorithm UACMS is increased by 13% on average compared with other algorithms.

To facilitate comparison, the MSE value of seven different algorithms in the dataset Brc was reduced to 40% of the original value, as shown in Figure 3. It can be seen from the figure that the algorithm proposed in this section has a dominant MSE value on the four datasets. In general, compared with other algorithms, the MSE value of the algorithm proposed is reduced by 0.83 on average, which shows certain advantages of UACMS. It is worth noting that Figure 3 shows that the MSE value of the method OF on Sol and renkou datasets is small, and the mean value of MSE on the 6 datasets is second only to UACMS. Since the MSE value reflects the tightness of objects in the cluster, the cluster generated by the method OF is relatively tight.

Figure 4 shows the F-score values of UACMS and the six comparison algorithms. Although CMS had the highest F-score in the dataset BrC, Eskin had the highest F-score in the dataset Sol, and UACMS had the best performance in the other four datasets and had the highest F-score mean of all datasets, which was about 13% higher than the mean of all comparison algorithms. Conversely, k-modes perform poorly on all datasets. This explains the reason for the k-modes' dependence on random initialization centers and lack of consideration for the interrelationships between attributes of objects.

Table 2 shows the runtime of the algorithm UACMS and the 6 comparison algorithms on 6 datasets. The algorithm UACMS has significant advantages on all datasets, and the average running time is improved by 11.32 minutes. Other six algorithms need more runtime along with the increase in the amount of dataset, but the runtime algorithm UACMS is not affected basically by the amount of dataset; this is because UACMS does not deal the original data, but the cluster centers of benchmark-scale dataset and the size of benchmark-scale dataset's cluster centers are far less than raw dataset. As CMS measures the similarity between objects, it needs to consider both the internal similarity of object attributes and the similarity between object attributes, which requires a relatively large amount of calculation, so the algorithm needs much more time, as shown in Table 2. The other five comparison algorithms are mature and efficient, especially k-modes, with short running time, but they have a common characteristic: with the increase in data volume, the execution time will increase accordingly. In particular, CMS and Eskin methods in the experiment are derived from the literature and were not optimized, so the operation efficiency was low.

In conclusion, through experiments, this section verifies that the proposed algorithm (UACMS) is superior to the other six algorithms in the clustering result indexes (NMI, MSE, and F-score) on most datasets. In addition, the biggest advantage of UACMS is that the runtime of UACMS is significantly shorter than that of the comparing algorithms, and it does not change much along with increasing data volume. This is because the UACMS deals with the knowledge on the benchmark-scale dataset rather than the original data. As a result, UACMS is available and efficient.

### 5.3. Downscaling

Figure 5 shows the NMI values of DSAL and 6 comparison algorithms on 6 datasets. Except for the dataset BrC, DSAL has the highest NMI value on the other five datasets, and the mean NMI value of DSAL on all datasets is about 19% higher than that of the six comparison algorithms. In contrast, the k-modes algorithm performs poorly in the experiment because, on the one hand, this method is built on the assumption that the attributes of the objects are independent, while the attributes of the objects in the experimental dataset are dependent; on the other hand, the k-modes algorithm randomly selects the cluster center during the execution, which leads to the randomness of clustering results. As the DSAL algorithm takes into account the interaction between different attributes, the clustering results have obvious advantages.

To facilitate comparison, the MSE values of six different algorithms in the dataset Brc are reduced to 40% of the original value, and the final MSE values of all algorithms are shown in Figure 6. It can be seen from Figure 6 that the MSE value of the algorithm DSAL is slightly unsatisfactory on the two datasets BrC and Titanic and is dominant on the three datasets except for renkou. However, the MSE value of the two algorithms HM and OF is slightly lower on the dataset renkou. The reason may be that there are fewer different attribute values in one attribute, which affects the performance of the relevant algorithm. Overall, the MSE value of DSAL in 3 of the 6 datasets was smaller than that of the comparison algorithm, with an average decrease of about 0.03. It shows that the compactness of cluster formed by the DSAL algorithm has a slight advantage over other comparison algorithms.

The F-score values of DSAL and the comparison algorithms are shown in Figure 7. It can be seen from Figure 7 that the DSAL has the highest F-score values in all the other five datasets except BrC, especially in dataset renkou, and the F-score value of this algorithm is about 46% higher than that of other methods. The average F-score of the algorithm OF is the least. The reason for the poor performance of the DSAL algorithm on the dataset BrC may be that the relationship between the attributes of the data objects is complex, and the designed function cannot fully reflect the relationship. However, overall DSAL's F-score improved by about 16% over the comparison algorithms. F-score takes both accuracy and recall rate into consideration. The larger the F-score, the better the clustering effect. Therefore, this algorithm has significant advantages in the real dataset renkou.

The runtime of the DSAL and the 6 comparison algorithms is shown in Table 3. Obviously, the CMS algorithm has the longest runtime on all datasets and needs further optimization. The algorithm DSAL is based on CMS, but the runtime is much shorter than the other six comparison algorithms, and the runtime is basically one order of magnitude shorter. This is mainly because the DSAL is related to the number of cluster centers of the benchmark-scale dataset, not amount of original data. Therefore, its running time is affected by the clustering results of bench-scale dataset, while the other six algorithms directly process the original data (after preprocessing), and their running time naturally increases gradually with the increase in data volume on the whole. On the dataset Titanic, the DSAL algorithm has less obvious advantage than k-modes, only using 0.27 seconds less, because it takes more time to solve the weight of cluster center using the kernel function Lanczos on this data. In particular, CMS and Eskin methods in the experiment were derived from the literature without any optimization, so the running time was relatively long. Since the running time is affected by computer hardware configuration and code optimization level, in addition, the running time in the comparison experiment is calculated under the specific environment, which is for reference only.

This section verifies that the proposed algorithm (DSAL) has obvious advantages in the external indicators (NMI and F-score) of clustering results on most datasets. Compared with the other algorithms, the DSAL's internal evaluation index MSE has a slight advantage. In addition, the biggest advantage of DSAL is that its runtime is significantly shorter than other algorithms, and it does not change much along with increasing data volume. This is because DSAL deals with the knowledge on the benchmark-scale dataset rather than the original data. Therefore, DSAL is available and efficient.

## 6. Conclusions

In this paper, a multiscale clustering algorithm based on coupling metric similarity is proposed, multiscale data mining is carried out for the multiscale nominal datasets with non independent and identical distribution, and a scale conversion method based on the benchmark-scale clustering results is proposed: the scale estimation method based on single chain UACMS and the scale estimation method based on Lanczos kernel. The experimental results show that proposed framework is efficient and effective on the datasets whose attributes are obvious multiscale properties.

In future work, we mainly focus on two aspects: (1) we are applying multiscale theory to frequent itemset mining and (2) the practical application of our study is worthy of attention, and we will consider applying multiscale clustering to collision detection and rule detection based on previous research studies.

## Figures and Tables

**Figure 1:** Overview of multiscale clustering.

**Figure 2:** NMI of UACMS vs. compared algorithms.

**Figure 3:** MSE of UACMS vs. compared algorithms.

**Figure 4:** F-score of UACMS vs. compared algorithms.

**Figure 5:** NMI of DSAL vs. compared algorithms.

**Figure 6:** MSE of DSAL vs. compared algorithms.

**Figure 7:** F-score of DSAL vs. compared algorithms.

**Algorithm 1:** Algorithm 1 Benchmark-scale clustering algorithm (BSCA).

**Algorithm 2:** Algorithm 2 Upscaling algorithm based on CMS (UACMS).

**Algorithm 3:** Algorithm 3 Downscaling algorithm based on Lanczos (DSAL).

**Table 1:** Properties of the datasets used for experimental analysis.

Dataset	*A*	*n*	*C*	Missing value
Zoo	16	101	7	No
Sol	35	306	18	Yes
Der	33	366	6	Yes
BrC	9	699	2	No
Titanic	5	1309	2	No
Renkou	4	5152	5	No

**Table 2:** Runtime of UACMS vs. compared algorithms (millisecond).

Dataset	CMS	HM	OF	IOF	Eskin	k-modes	UACMS
Zoo	44029	208	838	905	811	0266	57
Sol	2267711	1674	16931	18403	16551	3055	231
Der	3192750	2101	58454	29160	27747	1647	78
BrC	1784752	2642	44205	43379	52121	650	30
Titanic	1226818	2535	92365	88922	100047	0898	35
Renkou	10297337	136095	1305017	1318840	2270405	4389	50
Mean	3135566	24209	252968	249935	411280	1818	80

**Table 3:** Runtime of DSAL vs. compared algorithms (millisecond).

Dataset	CMS	HM	OF	IOF	Eskin	k-modes	DSAL
Zoo	43736	342	2071	982	809	294	15
Sol	2466067	8092	17349	18343	16583	3331	53
Der	3303631	3187	58247	59937	28071	1998	21
BrC	1760745	4057	43965	46712	53551	774	78
Titanic	1034446	11473	89457	97620	98447	966	703
Renkou	10028442	277075	1316525	1380572	2398618	5051	121
Mean	3106178	50704	254602	267361	432680	2069	165

## Data Availability

The data underlying the results presented in the study are included within the manuscript.
